The article "Application of Medical-Nursing-Assistance Integration Model Based on Theoretical Basis of Behavioral Psychology in Management of Children's ICU" was published in 2022. Journal: Comput Math Methods Med.

# Application of Medical-Nursing-Assistance Integration Model Based on Theoretical Basis of Behavioral Psychology in Management of Children's ICU

**DOI:** 10.1155/2022/1744357

**Published:** 2022-07-14

**Authors:** Yingying Jiang

**Affiliations:** Surgical Intensive Care Unit, Children's Hospital Affiliated to Zhejiang University School of Medicine, Hangzhou, 310000 Zhejiang Province, China

## Abstract

The children's intensive care unit is a closed management area with limited visiting time and no accompanying persons. It fails to systematically reflect and summarize the opinions and needs of the families of the children. The more critically ill the family members are, the higher the requirements for medical care. Good relationship between doctors, nurses, assistant, and patients can promote the rehabilitation of children's diseases and achieve the advanced medical model level of “seamless management and no loopholes.” In order to aid the complete intensive care process, it is vital to understand children's psychological and physical development based on children's behavioral psychology when the medical-nursing-assistance (MNA) integration model is used in the children's intensive care unit. Therefore, this paper has completed the following tasks: (1) the development status of the domestic and foreign MNA integration model in the quality management of children's intensive care units is introduced, and the MNA integration model based on the theoretical basis of behavioral psychology is proposed for the following article in children's intensive care. The effect evaluation system of room management provides a theoretical basis. (2) The principle of BP neural network is introduced, and the effect evaluation model of the integrated mode of MNA based on BPNN in the management of children's intensive care unit is constructed. (3) The relevant data collected are used to form an available data set for the model accuracy test. The experimental results show that, after the research in this paper, the BPNN model proposed in this paper is introduced into the MNA integration model to evaluate the effect of the management of children's intensive care units which is practical and effective.

## 1. Introduction

The children's ICU is a specific area equipped with a sufficient number of staff who have received special training and master the basic concepts, basic knowledge, and basic operating skills of critical medicine, including physicians, inspection technicians, nurses, and life assistants. Equipped with professional and technically necessary monitoring and treatment equipment to centralize the management, rescue, treatment, nursing, and rehabilitation of critically ill children, the purpose is to improve the rescue success rate of critically ill children and reduce mortality [1, 2]. The traditional medical model is the division of medical, nursing, and single-handling channels. The work is not completely connected, and there are loopholes and gaps. Real-time medical orders and auxiliary inspections are not implemented in a timely manner. The effect of medical order processing is not good.

It has drawbacks in the overall operation and management of children's ICU and cannot meet the management needs of children's ICU in comprehensive large hospitals, which has caused widespread concern in the medical community [3]. The requirements for treatment, nursing, and living needs of children's ICU work are higher than those of ordinary wards. Especially in the process of medical, nursing, and assistant shifts, it involves a wide range of areas. For example, children's ICU needs to understand children's psychological and physical development according to children's behavioral psychology during the medical and nursing process. Because children are in the primary development and growth stage of life, they are different from adults in behavior and psychology, so the medical and nursing processes are also different. Only a further understanding of children's psychology and behavior can contribute to the entire intensive care process [4]. Therefore, in the process of work, doctors, nurses, and life assistants need to be in close contact. The integration of MNA does not simply mean that doctors, nurses, and assistants work together, but a process of coworking in which the staff are independent, work division and cooperation, share information, help each other, promote each other, and share responsibilities; the patient's diagnosis and treatment, health education, and rehabilitation programs are jointly formulated by doctors, nurses, and patients after thorough communication. The integrated clinical nursing model of MNA builds a bridge between doctors, nurses, and life assistants, making the communication and cooperation between doctors, nurses, and assistants faster and more efficient. MNA are gradually subordinated to the implementation of active communication, mutual cooperation, and codominant transformation of medical and nursing staff. The integrated clinical nursing model of MNA is conducive to the formation of a positive cooperative attitude and promotes the increase of cooperative behaviors of MNA. At the same time, this mode makes the communication channels and methods between doctors, nurses, and assistants more smooth and effective and can quickly realize the exchange and information sharing of patient-related information, so that both doctors and nurses can more comprehensively understand the needs of patients and clearly understand the needs of patients. Changes in the condition are conducive to both medical and nursing parties to make correct decisions on clinical medical treatment and clinical nursing rehabilitation, thereby improving the overall quality of medical and nursing services. Studies have confirmed that the cooperative behavior of doctors, nurses, and assistants is an important factor that directly affects the quality of medical care, the relationship between doctors and nurses, patient health outcomes, and patient satisfaction [5–7].

MNA's integrated clinical nursing model requires nurses and assistants to incorporate the idea of doctor and patient participation in clinical nursing work such as nursing procedures and health education in order to achieve complementarity of specialised knowledge and professional skills among doctors, nurses, and assistants, as well as patients and caregivers, in order to obtain consistent and standardised scientific rehabilitation guidance and assistance from various perspectives. Some studies have proposed that positive medical-nursing cooperation is beneficial to changing the stereotyped image of patients and their families that nurses are subordinate to doctors. Patients and their families should give nurses enough trust and respect, which is an effective measure to improve the relationship between nurses and patients and the quality of nursing [8]. It is an inevitable trend to explore the integrated mode of medicine, nursing, and assistance. Doctors, nurses, and assistants all share the goal of providing a safe treatment environment and high-quality services to patients. The integrated model creates a positive relationship between nurses and patients, as well as between doctors and nurses. This study uses the integrated mode of MNA in the medical and nursing management of children's ICU to improve the safety of Chinese medicine prescriptions, the timely implementation of auxiliary inspections, and the timely follow-up of inspection reports. It can also improve nursing quality and safety, patient handover safety, infusion safety, and equipment management safety and improve the satisfaction of doctors, nurses, and assistants, with good results.

The following is the paragraph that organises the paper: the related work is found in Section 2. In Section 3, the methodologies used in the proposed work are examined.  Section 4 discusses the experiments and their outcomes. Finally, in Section 5, the research task is accomplished.

## 2. Related Work

With the transformation of the medical model to “biological-psychological-social medicine,” the traditional “dominant-subordinate” doctor-nurse relationship can no longer meet the needs of clinical work [9]. Under the background of the adjustment of medical relationship, “integration of medical and nursing,” as an advanced medical and nursing work mode, is widely carried out in various clinical departments and has achieved remarkable results. The integration of medical and nursing is essentially a localized concept, which is called “medical-nursing cooperation” internationally [10]. Since the concept of medical and nursing integration was put forward, its connotation has been continuously enriched and developed. Initially, some researchers believed that medical-nursing cooperation is essentially an interdisciplinary exchange, the core of which is that both nursing and nursing parties must participate in the entire process of patient assessment, decision-making, clinical goal formulation, and problem solving and share responsibilities [11]. In the 1950s, the UK and other European countries took the lead in implementing advanced nurse nursing activities and gradually formed a nursing model combining nurse and doctor services, which was conducive to the recovery of patients. Under this model, a benign teamwork model with reasonable division of labor, clear responsibilities, information sharing, close contact, and mutual cooperation has been formed between doctors and nurses. It is of positive significance to effectively improve the preoperative and postoperative anxiety and other emotions of patients, improve the patient's self-care ability, and improve the quality of life of patients [12]. This new model of healthcare cooperation is defined by the American Nursing Association as “a novel and trustworthy way of cooperation among healthcare workers that safeguards both sides' interests while attaining mutual goals.” But so far, many scholars have not formed a unified concept of the medical-nursing integration work mode, but they all include some common points. First of all, the medical-nursing integration work mode should be based on the mutual equality, respect, and trust of medical and nursing. On the premise of recognizing each other's professional knowledge and ability, through mutual communication and coordination, the specific method of participating in clinical decision-making by both medical and nursing parties is adopted, and there is shared responsibility for providing medical care to patients [13]. The medical-nursing integration work mode focuses on the joint participation and cooperation of both medical and nursing parties, mutual exchange of medical treatment and nursing, and joint provision of medical and nursing services for patients. Studies have shown that, compared with the traditional nursing mode in which both medical and nursing parties work separately, the integration of medical and nursing as an emerging work mode has greater advantages in improving the quality of medical and nursing services [14]. In the 1990s, reference [15] put forward four necessary conditions for medical cooperation, namely, ability, confidence, commitment, mutual respect, and trust. In 2003, the American Nursing Association (ANA) clearly defined healthcare cooperation as a process of trust-based and reliable cooperation between healthcare workers. At present, there is no consensus on the exact concept of medical and nursing integration. Although the views of various scholars include some common elements, their views are not exactly the same. Nevertheless, under the guidance of the medical-nursing integration model, the nursing quality of each clinical department has been significantly improved [16].

Reference [17] applied the medical-nursing integration model to the thyroid surgery clinic and established a collaborative group composed of specialist physicians and responsible nurses. And the medical staff are grouped according to their professional titles and ages, and each performs its own duties to ensure that patients are seamlessly connected in each diagnosis and treatment process. The study concluded that the medical-nursing integration model can effectively reduce the waiting time of outpatients and improve the service experience of medical staff. In 2013, the emergency department of a university-affiliated hospital introduced a medical-nursing integrated emergency patient-hospital process management model, which effectively solved the problems of low efficiency of emergency ward management and low efficiency of human-hospital contact. The work efficiency and satisfaction of front-line medical staff in the emergency department have been significantly improved [18]. As a result, this study uses a prospective research technique to assess the importance of routine nursing and integrated nursing care for patients, in order to create a more solid foundation for improving patient clinical nursing. The medical-nursing integration work paradigm has been widely utilised in the field of nursing to guide clinical nursing, nursing management, nursing research, and nursing education, with impressive outcomes. Reference [19] research shows that the integration of medical and nursing can improve the cooperation degree of medical and nursing work, the awareness rate of health education, and patient satisfaction. The research of reference [20] shows that the integrated medical and nursing work mode realizes the seamless connection between the transfer and handover departments, ensures the safety of patients, and improves the work efficiency. Reference [21] believes that the integration of medical and nursing has broadened the specialist knowledge of surgical nurses, improved the initiative and predictability of surgical cooperation, and is an effective method to improve the clinical practice ability of orthopaedic surgery specialist nurses. A university-affiliated hospital has successively carried out research on the medical-nursing integration cooperation model and believes that the medical-nursing integration work mode has achieved relatively good results in many aspects such as the synergy of the medical-nursing cooperation group, the improvement of the scientific research level of medical care, and the postoperative stress response of patients which have achieved relatively good results [22]

## 3. Method

### 3.1. Principle of BP Neural Network

#### 3.1.1. The Concept of BP Neural Network

The artificial neural network (ANN) is a computer information processing technique that can mimic the human brain. It is a frequently used machine learning algorithm with a lot of capability. In the ANN system, BPNN is a brilliant pearl. It mainly has the following characteristics:

1. Self-adaptation and self-learning: self-adaptive means that its own characteristics can adapt to changes in the environment and change accordingly. When the external environment changes, input new sample data into the neural network model for training, the model will automatically adjust the influencing parameters and mapping relationships during the training process, so that different input data can produce a desired output value within a specific range. Therefore, the neural network has stronger flexibility and adaptability than the expert system that uses a fixed model for calculation and is more similar to the operation law of the human brain
2. Nonlinearity problems in the real world are complex and nonlinear, and the human brain is also a nonlinear signal processing organization. Activating or inhibiting artificial neurons is essentially a nonlinear problem between processing data. The neural network reflects the data in the training samples to the connection weights to ensure that there is a nonlinear mapping relationship
3. The fault-tolerant BPNN has a wide distribution of nodes in the data storage process. When the input information is partially damaged, although the operating efficiency of the ANN will be moderately weakened, it will not lead to huge deviations in the operating results. This is very important in evaluation applications, because we often cannot be sure that every reference sample is absolutely correct
4. Computational parallelism and storage distribution inherent parallelism of BPNN enable each neuron to receive the input data accurately at the same time and then perform independent operation processing on the data and obtain the corresponding output result. Neurons in the same layer can perform operations at the same time and then output the results to the next layer for calculation processing through the transfer function. Therefore, the parallel computing of neural network can give full play to its advantages and improve the operation efficiency

#### 3.1.2. Structure of BP Neural Network

The data processing function of BPNN is closely related to the activity of neurons, how the neurons are connected, the size of the weights of the connections between neurons, and the maximum acceptance value of neurons.

1. Artificial neuron model: the neuron is the smallest unit of neural network, and its specific structure is shown in Figure 1, where *x*_*i*_(*i* = 1, 2, ⋯, *m*) is the input value of the neuron, *w*_*i*_(*i* = 1, 2, ⋯, *m*) represents the connection weight between the upper and lower levels of neurons, and *p* = *w*_*i*_ is the threshold of each layer node; if *x*_0_ = 1 is also regarded as the input value of the neuron, at this time, *w*_0_ is a special connection weight value, *f* is the transfer function, and *y* is the neuron output value; there are

(1) $$\begin{array}{c} y=f\left(\overset{m}{\underset{i=1}{\sum }}x_{i}w_{i}+p\right) \end{array}$$

(2) Hierarchical composition of BPNN

BPNN consists of an input layer, a hidden layer, and an output layer. The hidden layer may be from 1 to *n* layers, and the number of layers is mainly related to the complexity of the data to be processed.  Figure 2 shows a neural network with a double hidden layer structure. There are nodes at both ends of the three levels, and the connection weights between nodes are connected, and different nodes correspond to different thresholds. When there is a signal input, the input signal is first transmitted to the input layer and then passes through each hidden layer and output layer in turn, and finally, the result is obtained.

(3) Transfer function

The basic function of the transfer function of the BPNN is to activate the input and transform it into the output through the transformation of the transfer function. The transfer function must be differentiable from a mathematical point of view, otherwise it is meaningless. In the initial design of the model, the BPNN generally uses the sigmoid function as the transfer function of the hidden layer and the linear function as the transfer function of the output layer. At the same time, the sigmoid function can be divided into Log form and Tan form, which are selected according to whether the output value is negative. The specific form of the above transfer function is as follows:

Linear function

(2) $$\begin{array}{c} A=f\left(Wx+p\right)=Wx+p. \end{array}$$

Log-sigmoid function

(3) $$\begin{array}{c} f\left(x\right)=\frac{1}{1+{\text{e}}^{-x}}. \end{array}$$

Tan-sigmoid function

(4) $$\begin{array}{c} f\left(x\right)=\frac{1-e^{-2x}}{1+e^{-2x}}. \end{array}$$

#### 3.1.3. The Calculation Principle of BP Neural Network

BPNN is a self-correcting learning method. In the self-correction learning, each training sample corresponds to a learning signal, and many different learning signals jointly affect the output value. The network system regards the learning signal as the expected output. After the model is trained, the error between the expected output value and the actual output value will be obtained, and then, the network weights will be corrected many times according to the specific situation of the error. Through repeated self-learning and adjustment of the error, the model makes the error reach the preset local minimum value. At this time, the entire network forms a complete closed system. The size of the error can be measured by the mean square error between the output value of the output node and the expected value, thus forming a dependent variable with the input value as the independent variable, the connection weight as the correction coefficient, and the output value, by judging the size of the error. It is a function to evaluate the performance of the network, and the self-learning training of the network is transformed into the problem that the solution error falls into a minimum value.

The basic process of BPNN consists of two parts: forward propagation of learning signals and feedback propagation of output results. That is, the input value is processed layer by layer from the input layer, gradually approaching the output layer; the connection weights and node thresholds are corrected from the output layer.

1. The forward propagation process of the signal. Input value at hidden layer node:

(5) $$\begin{array}{c} \text{ne}{\text{t}}_{i}=\overset{M}{\underset{j=1}{\sum }}{\text{w}}_{ij}x_{j}+\theta \end{array}$$

Output value at hidden layer node *i*

(6) $$\begin{array}{c} y_{i}=\Phi \left(\text{ne}{\text{t}}_{i}\right)=\Phi \left(\overset{M}{\underset{j=1}{\sum }}w_{ij}x_{j}+\theta_{i}\right). \end{array}$$

The input value at node *k* of the output layer

(7) $$\begin{array}{c} \text{ne}{\text{t}}_{k}=\overset{l}{\underset{i=1}{\sum }}w_{ki}x_{i}+a_{k}=\overset{q}{\underset{i=1}{\sum }}w_{ki}\Phi \left(\overset{M}{\underset{j=1}{\sum }}w_{ij}x_{j}+\theta_{i}\right)+a_{k}. \end{array}$$

Input value at node *k* of the output layer

(8) $$\begin{array}{c} O_{k}=\varphi \left(\text{ne}{\text{t}}_{k}\right)=\varphi \left(\overset{q}{\underset{i=1}{\sum }}w_{ki}x_{i}+a_{k}\right)=\varphi \left[\overset{q}{\underset{i=1}{\sum }}w_{ki}\Phi \left(\overset{M}{\underset{j=1}{\sum }}w_{ij}x_{j}+\theta_{i}\right)+a_{k}\right]. \end{array}$$

(2) Error feedback propagation process: in error feedback propagation, first obtain the output result of the hidden layer in the output layer and then perform error analysis on the result; if the error is not within the expected range, adjust the output layer, hidden layer, and input weights and node thresholds between the layers; take the output results as input values; run toward the input layer; repeat the training for many times until the output results of the output layer are within the expected range; and then, end the operation. One-sample error function *E*_*p*_

(9) $$\begin{array}{c} E_{p}=\frac{1}{2}\overset{L}{\underset{k=1}{\sum }}{\left(T_{k}-O_{k}\right)}^{2} \end{array}$$

The multisample error criterion function *E*

(10) $$\begin{array}{c} E=\frac{1}{2}\overset{P}{\underset{p=1}{\sum }}\overset{L}{\underset{k=1}{\sum }}{\left(T_{k}^{P}-O_{k}^{P}\right)}^{2}. \end{array}$$

The following four formulas are the correction amount of the output layer weight Δ*w*_*ki*_, the correction amount of the hidden layer weight value Δ*w*_*ij*_, the correction amount of the output layer threshold value Δ*a*_*k*_, and the correction amount of the hidden layer threshold value Δ*θ*_*i*_. All of them are obtained by modifying the connection weights and node thresholds by the gradient descent method.

The formula for adjusting the weights of the output layer is as follows:

(11) $$\begin{array}{c} \Delta w_{ki}=-\mu \frac{\partial E}{\partial w_{ki}}=-\mu \frac{\partial E}{\partial y_{i}}\frac{\partial O_{k}}{\partial \text{ne}{\text{t}}_{k}}\frac{\partial \text{ne}{\text{t}}_{k}}{\partial w_{ki}}. \end{array}$$

The formula for adjusting the weights of the hidden layer is as follows:

(12) $$\begin{array}{c} \Delta w_{ij}=-\mu \frac{\partial E}{\partial w_{ij}}=-\mu \frac{\partial E}{\partial y_{i}}\frac{\partial y_{i}}{\partial \text{ne}{\text{t}}_{i}}\frac{\partial \text{ne}{\text{t}}_{i}}{\partial w_{ij}}. \end{array}$$

The formula for adjusting the threshold of the output layer is as follows:

(13) $$\begin{array}{c} \Delta a_{k}=-\mu \frac{\partial E}{\partial a_{k}}=-\mu \frac{\partial E}{\partial O_{k}}\frac{\partial O_{k}}{\partial \text{ne}{\text{t}}_{k}}\frac{\partial \text{ne}{\text{t}}_{k}}{\partial a_{k}}. \end{array}$$

The formula for adjusting the threshold of the hidden layer is as follows:

(14) $$\begin{array}{c} \Delta \theta_{i}=-\mu \frac{\partial E}{\partial \theta_{i}}=-\mu \frac{\partial E}{\partial y_{i}}\frac{\partial y_{i}}{\partial \text{ne}{\text{t}}_{i}}\frac{\partial \text{ne}{\text{t}}_{i}}{\partial \theta_{i}}. \end{array}$$

### 3.2. Determination of Network Parameters

The BPNN needs a large amount of prior data as support, and the calculation amount in the operation process is very huge. The Matlab scientific computing software launched by American MathWorks has powerful matrix computing capabilities, which greatly shortens the network training time. Using the neural network toolbox in Matlab can bring great convenience to users and related researchers. Users can directly call the functions in the toolbox to build a fully functional BPNN model. The neural network model in the Matlab toolbox mainly designs the input layer, the hidden layer, the output layer, the number of nodes in each layer, the connection weights and node thresholds, and the transfer function.

#### 3.2.1. Design of Input Layer and Output Layer

The selection of the number of nodes in the input layer and the output layer is determined by the actual situation. If the sample data is more complex, the more nodes are required to process the data. The number of nodes in the input layer is equal to the training dimension of the sample data, which can be the initial dimension or the dimension of the feature variable: the number of nodes in the output layer varies according to the network. In the classification network, select the number of categories, and in the simulation, select the output space dimension in the fit function in the fit network.

#### 3.2.2. Design of Hidden Layer

The design of the hidden layer mainly includes the design of the number of hidden layers and the number of nodes related to it.

*(1) Design the Number of Hidden Layers*. In the 1980s, Nielsen proved that a BPNN model with a single hidden layer can make a continuous function in any closed interval infinitely close to a regression value. Because a 3-layer BP design network with a single hidden layer is enough to complete any multidimensional mapping, double hidden layers are only needed to ensure the continuity of model learning when the function is discontinuous, so the neural network is mostly a single hidden layer or double hidden layers.

*(2) Design the Number of Hidden Layer Nodes*. The operation of the neural network is closely related to the number of hidden layer nodes. If there are not enough hidden layer nodes, the available mapping information will be insufficient, the error will be large, the fault tolerance rate will be low, and the sample recognition ability without self-learning will be weak, and it will be difficult to effectively complete the training; but if the number of hidden layer nodes is too large, it will be difficult to effectively complete the training. The structure of the neural network is complex, the number of iterations is increased, the operation efficiency is reduced, and the nonsalient content in the sample is input, which weakens the generalization ability. The generalization ability of ANN refers to the ability of neural network model to obtain correct output when inputting new data other than its training samples after completing multiple complete trainings. At present, the number of hidden layer nodes is often determined according to the personal experience of the model designer. Generally speaking, it is closely related to the number of input and output layer nodes, and the following formulas are usually used to determine the number of hidden layer nodes:

(15) $$\begin{array}{c} I=\sqrt{m+n}+b, \end{array}$$

where *b* is a constant value between 1 and 10, *n* is the number of nodes in the input layer, *I* is the number of nodes in the hidden layer, and *m* is the number of nodes in the output layer.

#### 3.2.3. Selection of BP Artificial Neural Network Algorithm

The BPNN has the advantages of simple operation, large scale of parallel processing data, less time-consuming, and high efficiency, making the BP algorithm one of the most widely used, stable, and perfect training algorithms at present. It essentially approximates the error of the output result to the extreme value of the expected range. However, when dealing with nonlinear issues, the gradient descent approach requires frequent modification of the connection weights and thresholds, which can result in a long training time, low learning efficiency, slow convergence speed, and an easy fall into the problem of local minimum range. Due to the above problems, the BP algorithm needs to be improved, and the commonly used methods are as follows:

1. Trainingdm additional momentum method: the additional momentum method makes the network consider both the effect of the error change and the influence of the error itself when modifying the connection weights. In the case where the additional momentum method is not used, the output value of the neural network may fall into the local minimum value, and after using the additional momentum method, the output value can skip these local values. This method uses the feedback propagation method to add a weight change value in the process to each old weight value to obtain a new weight value and repeat the training for many times to calculate the weight value change to achieve the minimum error and adjust the threshold which is the same as the above process
2. Trainingdx adaptive learning method: for a special and ambiguous problem, it is not easy to choose an appropriate learning rate. It is generally obtained through experience or experiments, and after starting training, the optimal learning rate will follow the training and changes with the progress. The network will fluctuate, and the output curve will oscillate if the learning rate is too high; if the learning rate is too low, the network will increase the training time, resulting in an increase in the number of convergence times and a slower network convergence rate, even if the network is stable. Therefore, it is hoped that by automatically adjusting the learning rate during the training process, the training efficiency can be kept the highest when the network is stable. The specific method of adjusting the learning rate is as follows: check the relationship between the connection weight and the error function at first. If the performance of the error function is reduced, it means that the learning rate is low and can be appropriately increased; if the performance of the error function is not reduced, it is improved; then, the learning rate should be reduced
3. Elastic algorithm: in the traditional BP algorithm, the activation function usually adopts the sigmoid function, which is characterized by the ability to convert any input value into an output value within a limited range. However, when the input value tends to infinity, the derivative will approach 0; that is, the gradient value will approach 0, and the network will stop modifying the weights. The elastic algorithm can effectively solve this problem. It only considers the positive and negative of the partial derivative, regardless of its specific value. The degree of weight update is determined by a predetermined independent value, and the direction of weight correction is determined by the sign of the partial derivative. In the process of two consecutive iterative derivations, if the sign of the partial derivative of the error function with respect to a certain weight does not change, the independent value will be increased. If the partial derivative changes, decrease the independent value. When the sign of the partial derivative remains the same in the continuous multiple iterations, it indicates that the direction of error correction is correct, and the workload of weight correction should be increased to improve the working efficiency of the neural network. Therefore, the elastic algorithm can significantly improve the speed and the convergence of the BP network

### 3.3. Evaluation Indicators for the Integration of Medicine, Nursing, and Assistance

Before constructing the evaluation indicators, the practical application of the medical-nursing-assistance integration model is introduced.

1. Before the implementation of the medical-nursing-assistance integrated model, the children's intensive care unit's morning shift mode is as follows: when the children's intensive care unit was handed over in the morning before the medical-nursing-assistance integrated model was implemented, the nursing work was the main content of the shift, and the doctor did not supplement it; instead, the doctor listened to the shift, focusing on the special situation of children at night, reviewing the imaging results and test results, and reviewing the medical history. Nurses get together to discuss the work of nursing. The doctors and nurses stagger the beds and rounds to avoid mutual interference, and then, the doctor issues a doctor's order, and the nurse immediately goes to process, execute the doctor's order, implement auxiliary examinations, and check abnormal examination reports. Nurses take over the shift in groups and pick up the beds, infusions, instruments, and equipment under their control. Life assistants assist nurses in daily care and receive visits from family members of children. Doctors, nurses, and assistants complete their duties within their respective responsibilities and conduct monthly self-examinations and quarterly inspections to evaluate the implementation of the core system of patient safety and nursing, supervision, and evaluation of the implementation of the nurse bed responsibility system and service satisfaction surveys
2. After the implementation of the integrated medical-nursing-assistance model, the shift mode of the children's intensive care unit: the nursing shift is the main priority, and the doctor on duty supplements the new admission, rescue, and abnormal reports of the children at night. Remind nurses what to focus on. Head nurses and department directors follow up on shifts involving patient safety, ward safety, and the opinions of patients' families to make rectifications. Medical assistants take part in discussions about complex situations, study documentation and materials, thoroughly analyze cases, and discuss any bottlenecks that arise. Conduct ward rounds for critically ill patients together, urge doctors and nurses to stay focused on their jobs, collaborate with medical care for multidisciplinary and critically sick patients, and put treatment and nursing measures in place. We should timely and correctly implement the emergency medical orders, implement the treatment plan as soon as possible, and feedback and track the treatment effect. For emergency auxiliary examination at the bedside, the nurse in charge of the bed assists the doctor to prepare medicines and supplies. Before going out, clean the respiratory tract; carry oxygen bags, first aid kits, warm appliances, and bed rails; and notify the transportation center to wait in the elevator. At the bedside, the mobile phone mobile core system can be used to check the inspection report in time and quickly, follow up the treatment of critical values, take special inspection results such as multi-drug-resistant bacteria, and take timely intervention measures, through joint participation in the discovery of nursing quality and safety, infusion safety, equipment safety hazards, the accuracy of infusion balance, pipeline medication arrangements, and equipment operation failure handling and other series of management. Everyone works together and participates in a working model that is both independent implementation and mutual cooperation. A small summary of daily shifts is posted on WeChat to facilitate the knowledge of all staff, regular medical-nursing-assistance communication meetings are held, family members are consulted in a timely manner, and the effect of the implementation of the integrated medical-nursing assistance model is summarized. The nurses' bed management responsibility system implements supervision and evaluation and service satisfaction survey
3. Indicators of observation and evaluation criteria are compared. The scale uses the patient safety and nursing core system implementation evaluation form to compare the number of defective cases of untimely execution of real-time doctor orders, untimely implementation of auxiliary inspections, poor doctor order processing, and untimely follow-up of inspection reports in children's intensive care units before and after the implementation of the medical-nursing-assistance integration model. Compared with the results of nursing projects, the quality of the bed unit was unsafe, the patient handover was incomplete, the infusion volume was incorrect, and the safety indicators of equipment were implemented. Investigate the satisfaction of doctors, nurses, and assistance services, and summarize the hospitalization and discharge feedback messages of the patient's family members

An evaluation method for the application effect of the integrated medical-nursing-assistance model based on the theoretical basis of behavioral psychology in the administration of children's critical care units was established based on the preceding descriptions, as shown in Table 1. The output is divided into three levels according to the input metrics.

## 4. Experiment and Analysis

### 4.1. Data Sources and Pretraining Processing

1. This study selects the data collected by a tertiary hospital from January 2016 to December 2017 in the implementation of the integrated medical-nursing-assistance model in the children's intensive care unit. The management of doctor's order processing effect, inspection report follow-up, bed unit environment safety, patient handover safety, infusion safety, and equipment safety management, using noncontemporaneous control, by comparing the integration before implementation (January 2014-December 2015) and implementation afterwards (January 2016-December 2017), the children's intensive care unit managed the safety of traditional Chinese medicine orders, the quality and safety of nursing, and the satisfaction of doctors, nurses, and assistants. 300 sets of data before and after implementation were obtained, respectively. Among them, 275 samples are used as the training samples of the neural network model, and 25 samples are used as the test samples of the neural network model
2. Usually, the input and output data of the neural network should be between 0 and 1. Since the model constructed in this paper does not meet such requirements, it is necessary to normalize the sample data before inputting it into the model. In this paper, the maximum and minimum method is used for normalization processing:

(16) $$\begin{array}{c} y=\frac{x-x_{\min}}{x_{\max}-x_{\min}}, \end{array}$$

where *x* is the sample data outside the interval [0, 1], *x*_min_ is the minimum number in the data sequence, *x*_max_ is the maximum number in the sequence, and *y* is the normalized value of the sample data *x*

### 4.2. Preliminary Training of the Model

#### 4.2.1. Model Construction Ideas

First, use all the information of the training samples, including the feature information of the training samples, to train the neural network. After the network adaptive learning is completed, input the features of the test samples to the trained network. The trained network will automatically analyze and predict and give the prediction of the effect level of the test sample predicted by the neural network model and compare it with the actual evaluation level of the corresponding test sample to judge the feasibility of the model.

#### 4.2.2. Initial Parameter Setting

The model is initially established by using the newff command in Matlab, and the initial parameter configuration of the network is set by default. The specific settings are shown in Table 2.

After the initial operation, it is found that the network output error of the model reaches the expected error range after 16 iterations, the time consumption is very short, and the error is also small, which shows that the network learning state is good.

#### 4.2.3. Model Test

The test of the model mainly starts from two aspects, the validity test and the accuracy test. As the name suggests, the validity test is to test the rationality of the model, such as whether the network convergence is reasonable and whether the model results are reliable, and the accuracy test is the correctness of the model, often measured by the error rate. The program's operating process can be used to reflect the validity test. The neural network's performance is poor when it runs slowly, has too many iterations, or has a big mean square error. As can be seen from the figure below, the indicators of the model established in this paper are relatively reasonable after the initial training. After 16 iterations of the model, the network output error reaches the expected error range, and the error value is 0.001625 within the effective range. The change process diagram is shown in Figure 3.

The accuracy test is mainly to test the gap between the input value of the neural network and the expected value, that is, the actual value of the test sample. The smaller the gap, the higher the accuracy. It is usually expressed by error or error rate, which is more suitable for the effect analysis of a single sample; you can also average multiple samples. Because this paper uses multiple samples to test the performance of the network, there is an error value for each sample data. We want the error rate to be as low as feasible; hence, this study uses a correct rate to assess the developed model's accuracy. It is the ratio of the number of times that the error rate between the actual value and the predicted value is within 10% of all the calculation results in the 275 training samples.

### 4.3. Optimization of the Model

Many parameters in the BPNN components, such as the number of hidden layers and their nodes, the selection of transfer functions, and the selection of training functions, will affect the final training results of the neural network. However, the specific selection of these parameters has not yet been accurately guided by the academic community, and more judgments are made through experience. Therefore, in order to ensure the accuracy and effectiveness of the neural network model, this paper decides that when the model is first constructed, the parameters that need to be determined are selected from the default parameters of the system, and then, the parameters of the model are adjusted one by one by controlling the parameter variables so as to finally determine a stable network model. The specific optimization process is as follows.

#### 4.3.1. Optimization of the Number of Hidden Layers

In this paper, a hidden layer is used in the initial training above, and a hidden layer is added below for training and result comparison. It can be seen from the test results that the accuracy of a single hidden layer is higher than that of a double hidden layer, so we do a more in-depth test on the basis of a single hidden layer. The test results are shown in Figure 4.

#### 4.3.2. Optimization of the Number of Hidden Layer Nodes

In this paper, 5 hidden layers are used in the initial training of the model, and integers around 5 are used as the number of hidden layers for testing. The test results are shown in Figure 5.

The data shows that when the number of hidden layer nodes is 5, the correct rate is high, so 5 is still selected as the number of hidden layer nodes.

#### 4.3.3. Optimization of Transfer Function

The commonly used transfer functions are logsig and tansig. The selection of transfer function has a great influence on the prediction result. The two transfer functions are tested, as shown in Figure 6.

The tabular data shows that the correct rate of the logsig function is higher, and the results of each correct rate are relatively stable, and the logsig function is still selected.

### 4.4. Analysis of Test Results

After combining the above model optimization, it is finally determined that the model has a single hidden layer structure with 5 hidden layer nodes, the transfer function selects logsig, and the training function selects trainlm. The running results of the optimized model are shown in Table 3.

It can be seen from the above table that the trained neural network can correctly predict the effect evaluation level, and the error is very low, which is a very significant level. At the same time, for the processing and analysis of 275 samples, the average time of BPNN is less than 2 s. The whole process is very convenient and much faster than the manual evaluation of evaluators. Applying performance evaluation is practical and remarkably efficient.

## 5. Conclusion

After the implementation of the medical-nursing-assistance integration model, the number of defects in the execution of real-time doctor's orders, the implementation of auxiliary inspections, the processing of doctor's orders, and the untimely follow-up of inspection reports in the children's intensive care unit decreased. Before the implementation of the integrated medical-nursing-assistance model, the children's intensive care unit mainly focused on the nursing work when the shift was handed over. The doctor did not supplement or provided little supplement, but after listening to the handover, the doctor focused on the special situation of the children at night. At this time, the content of the discussion is obviously related to the nursing shift, that is, the lack of a harmonious way and atmosphere of communication. The medical staff could not solve the problems encountered together. In order to avoid mutual interference, the doctors and nurses staggered the ward rounds, and then, the doctor issued a medical order without communicating the urgent needs to be dealt with in a timely manner. Irregular usage, inconsistent charging codes, etc. failed to communicate and urge improvement in a timely manner. There was a lack of effective communication in the real-time execution of medical orders and the safety of medical order execution. After the implementation of the integrated model of medical care and assistance, personnel supervision was strengthened and then improved. Working together can effectively prevent the occurrence of medical accidents and ensure patient safety. Improving and strengthening management and other countermeasures can effectively improve the quality of doctor's order execution and improve nursing quality and nursing safety. After running-in, communication, and implementation of the integrated model of medical and nursing assistance, the patient safety and nursing core system implementation evaluation is carried out through inspection, and real-time doctor's order execution and auxiliary inspection are displayed. The number of defects caused by untimely implementation, treatment of doctor's orders, and untimely follow-up of inspection reports is significantly lower than before the implementation. Therefore, this paper has completed the following work: (1) introduced the current state of the domestic and international medical-nursing-assistance integration model in the quality management of children's intensive care units and proposed a medical-nursing-assistance integrated model in children's intensive care units based on the theoretical foundation of behavioral psychology. The effect evaluation system of intensive care unit management provides a theoretical basis. (2) The principle of BPNN is introduced, and the effect evaluation model of the integrated mode of medical care and assistance based on BPNN in the management of children's intensive care unit is constructed. (3) The relevant data collected are used to form an available data set for the model accuracy test. The experimental results suggest that the BPNN model described in this study is realistic and effective when it is integrated into the medical-nursing-assistance integration model to evaluate the effect of the management of children's critical care units following the research in this paper.

## Figures and Tables

**Figure 1:** Neuron structure diagram.

**Figure 2:** BP model structure diagram.

**Figure 3:** Error change graph.

**Figure 4:** Test results when the number of hidden layers is different.

**Figure 5:** Test results of nodes in different hidden layers.

**Figure 6:** Different transfer function test results.

**Table 1:** Evaluation indicators for the integration of medicine, nursing, and assistance.

Index	Label
Execute medical orders in a timely manner	I1
Auxiliary inspections are implemented in a timely manner	I2
The doctor's order is very effective	I3
Follow-up of inspection reports in a timely manner	I4
Bed unit environmental safety	I5
Comprehensive patient handover	I6
Infusion balance is correct	I7
Instrument and equipment safety	I8
Patient satisfied with doctor	I9
Patient satisfied with nurse	I10
Patient satisfied with life assistant	I11

**Table 2:** Initial parameter settings.

Network parameters	Value or setting
Number of iterations	1500
Learning rate	0.15
Learning target	0.00005
Learning function	Trainlm
Hidden layer transfer function	Logsig
Number of hidden layer nodes	5

**Table 3:** Optimizing model run results.

Number	1	2	3	4	5	6	7	8	9	10
Accuracy	0.92	0.95	0.96	0.97	0.93	0.98	0.98	0.95	0.96	0.95

## Data Availability

The data sets used during the current study are available from the corresponding author on reasonable request.
